# Gait Recognition Based on the Plantar Pressure Data of Ice and Snow Athletes

**DOI:** 10.1155/2022/2982894

**Published:** 2022-07-30

**Authors:** Fengyu Wu, Xingyang Li, Wenyan Zhao, Bowen Ning

**Affiliations:** ^1^School of Sport Science of Harbin Sport University, Harbin, Heilongjiang 150008, China; ^2^Winter Olympic College of Harbin Sport University, Harbin, Heilongjiang 150008, China

## Abstract

The study of plantar pressure has become a research consensus in the field of biomechanics. The purpose of this paper is to study some lower limb movements in the daily activities of ice and snow athletes to obtain relevant data so as to carry out gait recognition analysis research. This paper selects the average foot pressure, forefoot foot pressure, front and rear foot pressure, foot pressure, toe pressure, 2–5 toe pressure, standing with eyes closed, *x*- and *y*-axes speed, foot length, foot width, and other actions of ice and snow athletes. Therefore, correlation analysis, work analysis, and curve fitting analysis were carried out on the joint motion in a single gait cycle. The collection and application of foot pressure and foot posture information are also analyzed. According to the plantar structure, the sole is divided into four parts. The maximum pressure point and coordinates of each part, the pressure center point, the ratio of the width and height of the sole of the foot, and so on are extracted as the haptic features of the gait. The experimental data shows that it can be seen that if the plantar area is divided in advance and the weight of each area is marked, whether standing, walking, or standing with one leg closed eyes can achieve better recognition results, and the accuracy rate is all more than 90 percent. The average recognition accuracy rate using the method of dividing four regions is only about 80%, and the accuracy rate of recognition using the method of dividing eight regions is 82%. It can be seen that the features extracted by the FCM model proposed in this paper contain more information of the plantar pressure image, and the accuracy rate is higher in the classification and recognition.

## 1. Introduction

At present, gait motion is often modeled by a series of multilink models. The model mainly calculates important motion information, such as displacement, velocity, and acceleration of the center of mass of each limb according to the angle changes of the ankle, knee, and hip joints. Among them, the angle change of the metatarsophalangeal joint is difficult to detect and only occurs during the foot contact, so it is often omitted in modeling. Although this move simplifies the calculation and analysis of the model, it also reduces the calculation accuracy of the model.

Gait recognition has the advantages of long-distance recognition, no active cooperation, nonintrusiveness, and difficulty in camouflage or concealment. However, gait recognition, as a new behavioral feature recognition technology, has shortcomings, such as low recognition rate and poor system robustness. The fusion of different features can improve the recognition rate of gait recognition. The gait recognition based on the fusion of vision and touch can improve the recognition rate and can recognize from a long distance without active cooperation. Research on gait recognition based on the fusion of gait vision and touch has important commercial value. It has good application prospects in important places, such as banks, parking lots, supermarkets, and airports.

The innovation of this paper lies in the following: (1) In order to reduce the feature dimension and improve the operation speed, the gait key frame is extracted. It selects double-support and single-support moments as key frame images. (2) According to the plantar structure, the sole is divided into four parts. The maximum pressure point and coordinates of each part, the pressure center point, the aspect ratio of the sole of the foot and other features are extracted. (3) A gait recognition algorithm is proposed, which integrates lower limb angle features and plantar pressure distribution features on the feature layer. Feature layer fusion is performed on the features to form a new feature vector.

## 2. Related Work

Falls are common accidents that can result in bruising and serious injury. The purpose of Niu et al.'s research is to gain an in-depth understanding of the feasibility of data mining techniques to intervene in tripping-related occupational safety problems. Although power spectral density (PSD) and support vector machine (SVM) were used to analyze the characteristics of plantar pressure distribution during limping and normal gait [1], the characteristics of plantar pressure during tripping and the differences between tripping and normal gait are still unclear. It becomes more important to use gait to detect whether a fall will occur. Lee et al. conducted experiments on four types of falls and eight activities of daily living using an integrated sensor system of an inertial measurement unit and a plantar pressure measurement unit simultaneously. The results show that the fall detection algorithm has a fall detection accuracy of 95% or higher, with an average lead time of 317 ms [2]. Although the threshold method and decision tree method are used to collect data, their application is not very extensive. Human gait recognition is important for controlling the exoskeleton and enabling smooth transitions. To accurately control exoskeleton motion, Wang et al. developed a multisensor fusion gait recognition system. The results show that the SVM algorithm has a high recognition rate, with an average recognition accuracy of 96.5% [3]. Although the system obtains the plantar pressure and acceleration signals of the human leg, there are still errors. Chen et al. proposed a whole-body exoskeleton gait phase recognition method using only joint angle sensors, plantar pressure sensors, and inclination sensors [4], but it was not trained using phase-labeled gait data.

Evolutionary decision fusion has applications in biometric authentication and verification. Kumar et al. proposed a new method based on decision fusion to solve [5]. Although gait data is simultaneously recorded using motion sensors and visible-light cameras, the issue of a better approximation of the underlying search strategy is not addressed. Gait recognition is one of the most important technologies in application fields, such as video surveillance, human tracking, and medical systems. Wang et al. presented a new Gabor wavelet-based gait recognition algorithm. Experimental results show that the proposed gait recognition algorithm is robust in general and has higher recognition accuracy compared with existing methods [6]. Human natural walking and topological analysis has its own unique key characteristics. It can identify when other biometrics are not visible. The purpose of Sayed is to draw attention to a simple and novel feature extractor for gait recognition based on deep learning methods [7]. Although the proposed gait recognition method achieves profound results in terms of training/validation accuracy and mean squared error, the experimental results do not have competitive performance.

Combined with the development status and difficulties of gait recognition, the development trend of gait recognition mainly has the following three directions. From the perspective of vision, it is necessary to solve the problems of background modeling and motion segmentation in complex environments, human occlusion and occlusion of moving objects, multiview recognition, and the establishment of larger-scale databases. From the haptic point of view, it is necessary to propose features and recognition algorithms that can better characterize the nature of gait motion. From the perspective of data fusion, we can study the fusion of different features in gait, the fusion of gait, and other biological features, such as the fusion of gait and face.

## 3. Current Status and Methods of Gait Recognition from Plantar Pressure Data

### 3.1. Biometric Technology

Biometrics combines existing advanced technologies, such as biometric principles, acoustics, and computer technology, to confirm identity through biometric data [8]. Biometrics can be used for identification, but no biometrics is perfect, and different biometrics have different characteristics and uses. Common biological characteristics are shown in Figure 1.

As shown in Figure 1, fingerprint recognition realizes recognition by comparing the details of fingerprints and has the characteristics of high recognition rate, fast recognition speed, reliability, and uniqueness. While fingerprint recognition is a physical contact, fingerprints are easily worn and forged [9]. Facial recognition achieves recognition by analyzing and comparing the visual features of the face. It is noncontact and noninvasive. But since the human face is easily affected by age, facial expressions, makeup, and so on, it is easy to be hidden or camouflaged, so the recognition effect is very good. Iris recognition is characterized by the texture of the human iris, which is highly stable and unique. It can be used for noncontact data collection within a certain distance. However, there are problems, such as the inability to collect data for the visually impaired and the high cost of collection equipment [10]. Palmprint recognition is based on detailed information, such as lines and textures of palm images. However, physical contact is also required during data collection, and the dry humidity of the hands has a greater impact on data collection. Voice recognition is through the matching of voices for identification without physical contact. However, it is greatly affected by environmental noise, and the recognition rate is low [11]. Handwriting recognition is to compare the detailed information, such as gestures and pressure of the test sample, with the database sample to identify the authenticity of the handwriting sample, which is easy to be accepted by people, but with the growth of experience, changes in lifestyle and personality, signature, and so on will also change.

### 3.2. Human Gait Basis

#### 3.2.1. Gait Recognition of Plantar Tactile Features

Gait recognition based on plantar tactile features involves a variety of disciplines, such as sports biomechanics, human anatomy, computer science, and technology. Its general process is shown in Figure 2.

As shown in Figure 2, gait tactile information can be divided into macroscopic information and microscopic information. Human walking trajectory and ground reaction force belong to the category of macroscopic information. The pressure distribution in each distribution area of the sole belongs to microscopic information. Human gait roughly conforms to the law of bipedal motion. However, different people's gait movements have their own characteristics and differences, such as the difference in cycle and step length. Therefore gait is also considered unique [12]. In conclusion, the fields of medicine, psychology, and biomechanics have demonstrated that gait is unique. This provides a strong scientific basis for the study of gait recognition.

#### 3.2.2. Division of Gait Phases

Alternating repetitions of the same type of basic leg and foot movement is called the human gait, which is a cyclic movement phenomenon. For faster analysis and understanding of this periodic motion process, it is necessary to accurately describe the complete gait cycle through gait timing [13]. The correct division of gait stages describes the intrinsic functional significance of each joint in the body. This positively contributes to the analysis of gait. In general, physiological events that divide gait phases are critical actions. A schematic diagram of a complete gait cycle is shown in Figure 3.

As shown in Figure 3, the human gait cycle can generally be divided into seven separate executions: initial contact, load response, intermediate support, final support, initial swing phase, intermediate swing phase, and final swing phase. There are three phases: contact phase, support phase, and swing phase. A walking cycle from the grounding of the heel on one side to the grounding of the heel on the same side is called a walking cycle, which consists of a support phase and a swing phase. The support phase refers to the period when the foot is in contact with the ground, including 5 periods of heel contact, sole contact, mid-support period, heel clearance, and toe clearance; swing phase is the period when the foot leaves the ground. It consists of two periods, the middle swing period and the deceleration period. In a normal walking cycle, the support phase is 60%, of which about 10% is a double-support phase, and the swing phase is 40%. These percentages are measured by normal people walking at a comfortable pace, and these percentages can vary widely as walking speed changes. Increasing walking speed increases the time in the single-support phase and shortens the time in the dual-support phase. When walking, the center of gravity of the body should move up and down by about 5°, and the pelvis should be rotated back and forth by about 8°. The maintenance of normal gait should be 30° of hip flexion forward and 10° of backward extension; full extension of the knee joint, 60° of flexion; 20° of plantar flexion of the ankle joint, and about 15° of dorsal extension.

### 3.3. Fuzzy *C*-Means Clustering Algorithm

Although the foot pressure feature vector extracted by SVD and PCA contains the feature information of human gait motion, the spatial distribution of the corresponding feature points is not intuitive. Therefore, it needs to be clustered and divided, and the walking state of the human body should be identified from the division results [14]. Fuzzy *C*-means (FCM), as a clustering method, measures the degree of each data point belonging to different clusters by the degree of membership. The corresponding fuzzy clustering characteristics just meet the fuzzy requirements of gait motion classification.

Assuming that the walking process of a normal person can be divided into two feet standing still, single foot support (left foot), double foot support (left foot behind and right foot in front), single foot support (right foot), and double foot support (right foot behind left foot). In these five typical states, the fuzzy group takes *c* = 5, and the corresponding objective function and constraints are as follows:

Objective function:

(1) $$\begin{array}{c} \min J=\sum_{i=1}^{5}\sum_{j=1}^{n}u_{ij}^{m}{\left\|p_{j}c_{i}\right\|}^{2}=\sum_{i=1}^{5}\sum_{j=1}^{n}u_{ij}^{m}u_{ij}^{m}{\left\|p_{j}-c_{i}\right\|}^{2}. \end{array}$$

Restrictions:

(2) $$\begin{array}{c} \sum_{i=1}^{5}u_{ij}=1,\;\forall j=1,\ldots ,n. \end{array}$$

The objective function and constraints are linked so as to realize the transformation to the unconditional extreme value problem; namely,

(3) $$\begin{array}{c} \min J{}^{\prime }=\sum_{i=1}^{5}\sum_{j=1}^{n}u_{ij}^{m}{\left(p_{j}-c_{i}\right)}^{2}+\sum_{j=1}^{n}\lambda_{j}\left(\sum_{i=1}^{5}u_{ij}-1\right). \end{array}$$

The partial derivative of the variable *c*_*i*_ in formula (3) has

(4) $$\begin{array}{c} \frac{\partial J^{\prime }}{\partial c_{i}}=\sum_{i=1}^{5}\sum_{j=1}^{n}\frac{\partial u_{ij}^{m}{\left(p_{j}-c_{i}\right)}^{2}}{\partial c_{i}}-\frac{\partial }{\partial c_{i}}\sum_{j=1}^{n}\left(\sum_{i=1}^{5}u_{ij}-1\right). \end{array}$$

Since ∑_*i*=1_^5^*u*_*ij*_=1,  ∀ *j*=1,…, *n*, that is,

(5) $$\begin{array}{c} \frac{\partial }{\partial c_{i}}\sum_{j=1}^{n}\lambda_{j}\left(\sum_{i=1}^{5}u_{ij}-1\right)=0. \end{array}$$

Formula (5) is substituted into formula (4), and it is set to 0 to have

(6) $$\begin{array}{c} \frac{\partial J^{\prime }}{\partial c_{i}}=\sum_{i=1}^{5}\sum_{j=1}^{n}\frac{\partial u_{ij}^{m}{\left(p_{j}-c_{i}\right)}^{2}}{\partial c_{i}}=-2\sum_{i=1}^{n}u_{ij}^{m}\frac{\partial \left(p_{j}-c_{i}\right)}{\partial c_{i}}=0. \end{array}$$

After arranging the transfer items, the solution can be obtained as follows:

(7) $$\begin{array}{c} c_{i}=\frac{\sum_{j=1}^{n}u_{ij}^{m}p_{j}}{\sum_{j=1}^{n}u_{ij}^{m}}. \end{array}$$

Then, take the partial derivative of the variable *u*_*ij*_ in formula (3), which has

(8) $$\begin{array}{c} \frac{\partial J^{\prime }}{\partial u_{ij}}=\frac{\partial }{\partial u_{ij}}\sum_{j=1}^{n}\sum_{i=1}^{5}u_{ij}^{m}{\left(p_{j}-c_{i}\right)}^{2}+\frac{\partial }{\partial u_{ij}}\lambda_{j}\left(\sum_{i=1}^{5}u_{ij}-1\right). \end{array}$$

That is, for there is

(9) $$\begin{array}{c} u_{ij}={\left(\frac{-\lambda_{j}}{m{\left(p_{j}-c_{i}\right)}^{2}}\right)}^{-1/m-1}. \end{array}$$

Formula (9) is substituted into formula (2); it has

(10) $$\begin{array}{c} {\sum_{i=1}^{5}\left(\frac{-\lambda_{j}}{m{\left(p_{j}-c_{i}\right)}^{2}}\right)}^{1/m-1}=\frac{{\left(-\lambda_{j}\right)}^{1/m-1}}{\sum_{i=1}^{5}{\left(m{\left(p_{j}-c_{i}\right)}^{2}\right)}^{1/m-1}}=1,\;\forall j=1,\ldots ,n. \end{array}$$

That is, (−*λ*_*j*_)^1/*m*−1^=∑_*i*=1_^5^(*m*(*p*_*j*_ − *c*_*i*_)^2^)^1/*m*−1^, which is substituted into formula (9) to get the solution as follows:

(11) $$\begin{array}{c} u_{ij}=\frac{\sum_{i=5}^{5}{\left(m{\left(p_{j}-c_{i}\right)}^{2}\right)}^{1/m-1}}{{\left(m{\left(p_{j}-c_{i}\right)}^{2}\right)}^{1/m-1}}={\left(\frac{{\left(p_{j}-c_{i}\right)}^{2}}{\sum_{i=1}^{5}{\left(\left(p_{j}-c_{i}\right)\right)}^{2}}\right)}^{1/m-1}. \end{array}$$

So far, the operation formula of the core iteration parameters in the FCM algorithm is obtained.

### 3.4. Evaluation of Clustering Effect

After the feature points are clustered and divided into *b* by the FCM algorithm, the validity and quality of the division results need to be quantitatively evaluated [15]. Generally, there are two types of evaluation and measurement methods for clustering effect, one is internal evaluation method; the other is external evaluation method. The difference between the two is that the external clustering effect evaluation method has the correct sample clustering result label as a reference; that is, the clustering label of the sample point is given in whole or in part. Thus, the actual clustering results can be compared with the given clustering labels, and a reliable clustering effect evaluation can be obtained [16]. However, for the samples to be clustered, the correct clustering labels are often difficult to obtain. The internal clustering effect evaluation rule has no clustering labels for reference. It is mainly based on some relative mathematical indicators as the evaluation basis. Therefore, compared with the external method, it has the characteristics of poor reliability but strong adaptability [17].

If the result of clustering can be divided into *n* cluster subsets according to clusters, that is, there is *C* = {*C*1, *C*2,…, *Cn*}, then there are the following parameter definitions:

(12) $$\begin{array}{c} \text{avg}\left(C\right)=\frac{2}{\left|c\right|\left(\left|c\right|-1\right)}\sum_{1\leq i\leq j\leq |C|}\text{dist}\left(x_{i},x_{j}\right). \end{array}$$

Among them, avg(*C*) is the average distance between samples obtained by summing and averaging the Euclidean distances of the samples in the aggregate taxonomic cluster *C*.

(13) $$\begin{array}{c} \text{diam}\left(c\right)=\underset{1\leq i\leq j\leq \left|C\right|}{\max}\text{dist}\left(x_{i},x_{j}\right). \end{array}$$

Diam(*C*) is the farthest distance of the obtained samples after taking the maximum distance of the samples in the aggregate taxonomic cluster *C*:

(14) $$\begin{array}{c} d_{\min}\left(C_{i},C_{j}\right)=\underset{x_{i}\in c_{i},x_{j}\in c_{j},}{\min}\text{dist}\left(x_{i},x_{j}\right), \end{array}$$

where *d*_min_(*C*_*i*_, *C*_*j*_) is the closest sample distance between the two clusters of aggregate taxonomic cluster *C*_*i*_, *C*_*j*_.

(15) $$\begin{array}{c} d_{\text{cen}}\left(C_{i},C_{j}\right)=\text{dist}\left(\mu_{i},\mu_{j}\right), \end{array}$$

where *d*_cen_(*C*_*i*_, *C*_*j*_) is the distance between the cluster center points of each clustered classification cluster *C*_*i*_, *C*_*j*_; *μ*_*i*_ is the cluster center point of each clustered classification cluster; and dist is the distance function between two points. The relevant evaluation index is the DB index (Davies–Bouldin Index, DBI):

(16) $$\begin{array}{c} \text{DBI}=\frac{1}{k}\sum_{i=1}^{k}\underset{i\neq j}{\max}\frac{\text{avg}\left(c_{i}\right)+\text{avg}\left(c_{j}\right)}{\text{dcen}\left(\mu_{i},\mu_{j}\right)}. \end{array}$$

A smaller DBI index means a smaller distance between classes and a larger distance between classes.

Dunn Index (DI):

(17) $$\begin{array}{c} \text{DI}=\underset{1\leq i\leq k}{\min}\left\{\underset{i\neq j}{\min}\left(\frac{d_{\min}\left(C_{i},C_{j}\right)}{\max\text{ diam}{\left(C_{l}\right)}_{i\leq l\leq k}}\right)\right\}. \end{array}$$

A larger DI index means a larger distance between classes and a smaller distance between classes.

### 3.5. Gait Motion Symmetry

For the symmetry analysis of human gait motion, it can be converted into a similarity analysis of the movement trends of the left and right leg joints during walking [18]. Now suppose that the motion parameters of the left and right leg joints are two groups of continuously changing random signals *x*(*t*) and *y*(*t*), and the cross-correlation function of the two is

(18) $$\begin{array}{c} R_{xy}\left(\tau \right)=\int_{-\infty }^{+\infty }x\left(t\right)y\left(t+\tau \right)\text{dt}=x\left(t\right)*y\left(t+\tau \right), \end{array}$$

that is, the convolution of the two signals. If *R*_*xy*_(*τ*) reaches the maximum value at *τ*=*τ*_*d*_, it indicates that the signal *x*(*t*) and *y*(*t*) have the greatest correlation after the phase shift *τ*_*d*_, and the similarity of the signal change trend is the highest [19]. However, the actual sampling of joint motion parameters is discrete signal, and in one gait cycle (1.2 s), there are *N* = 72 sampling data in total. For each sampling period *T* = 1.2/72 = 1/, the corresponding normalized cross-correlation function is

(19) $$\begin{array}{c} r_{xy}\left(k\right)=\frac{\sum_{i=1}^{k}\left(x_{i}-\bar{x}\right)\left(y_{i+n-k}-\bar{y}\right)\sum_{i=k+1}^{N}\left(x_{i}-\bar{x}\right)\left(y_{i-k}-\bar{y}\right)}{\sqrt{\sum_{i=1}^{N}{\left(x_{i}-\bar{x}\right)}^{2}}\sqrt{\sum_{i=1}^{N}{\left(y_{i}-\bar{y}\right)}^{2}}}. \end{array}$$

Among them, *r*_*xy*_(*k*) ∈ [−1, 1] is the correlation coefficient obtained after the correlation degree of the two signals to be analyzed is analyzed and then normalized [20]. It takes the rotation angle changes of the left and right leg joints as two sets of motion sampling data, and substitutes them into formula (19) for calculation and analysis. The results are shown in Figure 4.

As can be seen from Figure 4, when *k* = 36, the maximum cross-correlation coefficient of the left and right leg ankle joint movements is 0.878. That is, after the left and right ankle joint angles are shifted in time by *τ* = *T*·*k* = 0.6 s, the movement trend is highly correlated. Similarly, it can be calculated that the torques of the joints of the left and right lower limbs also have similar correlation characteristics. The abovementioned high correlation of left and right leg joint motion supports the idealized assumption of gait motion in the paper [21, 22]. That is, the left and right leg gait is a symmetrical planning movement. The establishment of this gait symmetry assumption simplifies the corresponding research work. It makes it possible to learn the complete gait movement law from the movement of the unilateral lower limb through mirror symmetry. And the correlation degree analysis of the left and right lower extremity movements can also be applied to the analysis of clinical pathological gait, such as quantitative evaluation of the recovery degree of the patient's walking ability [23].

### 3.6. Abnormal Gait and Analysis of Common Ice and Snow Athletes

After gait recognition of plantar pressure data, it is found that ice and snow athletes have common abnormal gaits, as follows:

1. Foot inversion: Foot inversion is the most common pathological gait, more common in patients with upper motor neuropathy, often combined with foot drop and toe curling. When walking, the main part of the foot touching the ground is the anterolateral edge of the foot, especially the base of the fifth metatarsal. There is often pain in the load-bearing part, which leads to instability of the ankle joint and affects the balance of the whole body. Compensatory flexion of the hip joint may occur, and the ability to clear the ground during the swing phase of the affected limb is reduced. Associated muscles include tibialis anterior, posterior tibialis, flexor digitorum longus, gastrocnemius, soleus, extensor pollicis longus, and peroneus longus.
2. Foot valgus: It is more common in children or young patients with immature skeletal development (e.g., cerebral palsy), which manifests as the foot tilts laterally when walking, and the medial side of the supported foot touches the ground, and may have toe flexion deformity. When walking, the center of gravity of the body mainly falls on the anterior and medial ankles. Relevant muscles include peroneus longus, peroneus brevis, flexor digitorum longus, gastrocnemius, and soleus.
3. Knee hyperextension: Knee hyperextension is very common, but it is usually a compensatory change, and it is more common in the early stage of support. Weakness of one knee can lead to compensatory hyperextension of the contralateral knee; flexor toe spasm or contracture leads to hyperextension of the knee; knee hyperextension compensation for knee collapse gait; spasm of extensor muscles; and land in front of the knee's center of gravity, pushing the knee back to maintain balance.
4. Short-leg gait: When the affected limb is shortened by more than 2.5 cm, the ipsilateral pelvis descends when the side touches the ground, causing the ipsilateral shoulder to tilt and descend, and the contralateral swinging leg is overflexed at the hip and knee joint and at the ankle joint. If the shortening exceeds 100px, the shortened side lower limbs are walked on the toes, and the gait is collectively referred to as the short-leg gait.
5. Gluteus maximus gait: The gluteus maximus is the main hip extensor and spinal stabilizer. Control the center of gravity forward when hitting the ground. If the gluteus maximus is weak, the heels often use force to protrude the waist forward so that the gravity line falls behind the hip joint, forming a gluteus maximus gait with chest and abdomen raised.
6. Gluteus medius gait: In the early and middle stages of stance, the pelvis moves down to the affected side by more than 5°, the hip joint is convex to the affected side, and the patient's shoulders and waist appear compensatory scoliosis to increase pelvic stability. The lower limb on the affected side is relatively long, so the knee and ankle flexion is increased during the swing phase to ensure ground clearance. The typical gait feature is the duck step.

## 4. Gait Recognition Experiment of Ice and Snow Athletes' Plantar Pressure Data

### 4.1. Database Situation and Data Preprocessing

The database of this paper includes static data collected while standing still on one leg with eyes closed and data of walking at three different speeds. The total number of them was 35, including 29 males and 6 females. Males weigh between 55 kg and 75 kg and are about 168–178 cm tall. Females weigh between 40 kg and 55 kg and are about 158–168 cm tall. Both men and women were between the ages of 20 and 28, and data was collected on both their left and right feet at the same time.

For the data in the static database, from the collected plantar pressure data of 35 people, each person selects 10 frames with relatively stable pressure values for the left and right feet as training samples, and 3 frames as test samples; the training samples are 1000 soles' pressure images (500 left foot, 500 right foot), and the test sample was 300 plantar pressure images (150 left foot, 150 right foot). According to the theory of footprint analysis and inspection, the plantar pressure and gait analysis system divides the plantar surface into ten parts for collection, which are the great toe area (T1), the 2–5 toe area (T2–5), the first plantar area (M1), second plantar area (M2), third plantar area (M3), fourth plantar area (M4), fifth plantar area (M5), arch area (MF), medial heel area (HM), and heel area lateral zone (HL). After the plantar pressure data collection is completed, the effective value of their pressure data is saved. For the data in the dynamic database, key frames should be selected before extracting the plantar pressure information for gait recognition. Because the distribution of plantar pressure is different for the same person every time they walk, but the frame with the largest total pressure has more complete footprint information and stable changes in pressure value, the plantar pressure used to characterize a walk is representative. Therefore, the frame with the maximum total plantar pressure is selected as the key frame data.

### 4.2. Multisensor Configuration

In order to obtain more comprehensive gait foot pressure information, it refers to human anatomy and foot pressure distribution. The human foot is divided into regions, and flexible pressure measurement units are placed in these regions to form a multisensor foot pressure detection system. In a gait cycle, the statistical variation of pressure signals in different regions is shown in Figure 5.

As shown in Figure 5, in a complete gait detection cycle, affected by the special ground contact form of the foot, the pressure sensor of the multipoint array can only collect the foot pressure signal of the corresponding local area in different gait periods. For example, sensors in the heel area can only record pressure signals during gait touchdown. When the heel is off the ground, the pressure signal cannot continue to be effectively collected, and the sensors in other positions have a similar situation. At the same time, the overlap and redundancy between signals also increase the burden on the detection system in data transmission, processing, and storage. Therefore, it is necessary to optimize the configuration of the pressure sensors in the eight regions of the sole of the foot. In this way, with the optimal sensor array position and the minimum number of sensors, the maximum amount of information can be obtained from the limited collected signals, and finally the ideal detection result can be obtained.

The data of different people's walking measurements and even the same person's multiple walking measurements are not the same, but the overall trend and the approximate range of joint angles are similar. By observing the contrast signal situation, it is possible to find the salient features of different synchrony when walking. The angle signal is discussed below in two cases, and the eigenvalues that can achieve the purpose of differentiation are obtained.

#### 4.2.1. Angle Information of Joints

It combines the obtained data with the division of the gait cycle in the typical lower limb movement gait, extracts the joint angle of a gait cycle, and normalizes the cycle. The angles of the three joints in the five gaits were compared, and the ordinate represented the joint angle, and the abscissa represented the time percentage of the gait cycle. The single-cycle hip joint angles for the five gaits are shown in Figure 6.

It can be seen from Figure 6 that the angle change of the hip joint is only negative when walking on flat ground, and all other gaits are all positive. The curves for going up stairs and going uphill are similar, just moving relative to time. That is, the time to reach the maximum value is different. Likewise, the curves for descending stairs and descending slopes are similar, but the magnitude of the change is different.

#### 4.2.2. Angle Information of Gait

On the basis of analyzing the angle information by joints, the three-joint angle characteristics of the five gaits are studied in detail. It obtains the three-joint angle information of hip, knee, and ankle in five gaits: walking on level ground, descending stairs, descending slope, ascending stairs, and ascending slope, respectively. The walking gait cycle is divided into the early support period, the middle support period, the support end period, and the swing period. The joint angle curve changes under the five gaits are shown in Figures 7 and 8.

As shown by the changes in knee joint angles in Figures 7 and 8, the five gaits changed significantly during the swing phase. The curves of walking on level ground, going down stairs, and going downhill are similar, and the curves of going up stairs and going uphill are similar. The difference between the five gaits is the amplitude and the time of the peak. The change of ankle joint angle is mainly concentrated in −20°∼−40°, and the change is the most complicated. At the beginning of the gait cycle, the angle of dorsiflexion was the largest in uphill, followed by upstairs. The angle value of walking on level ground and descending slope is close to 0°, and descending stairs is plantar flexion. The change is also more pronounced during the swing period.

### 4.3. Plantar Pressure Signal Processing

For the plantar pressure signal that outputs high and low levels, the signal is normalized. It sets the value to a high or low level of 0 or 0.5, and the foot pressure is represented by a solid line. The heel is indicated by a long dashed line. When both the ball and heel pressures are 0, the gait is in the swing phase. When there is pressure on the heel and the pressure on the sole of the foot is 0, it means that the gait is in the early stage of support. When there is pressure on both the ball of the foot and the heel, the gait is in mid-support. When there is pressure on the ball of the foot and the pressure on the heel is 0, it means that the gait is in the end of support. This is used as a criterion for dividing the gait cycle. The set gait phases are represented by numbers, where 2 is the prestance phase, 3 is the mid-stance phase, 4 is the end-stance phase, and 5 is the swing phase. The obtained plantar pressure signal, the normalized plantar pressure signal, and the ladder diagram representing the gait stage are shown in Figure 9.

As shown in Figure 9, the sensor signals for the five gaits are filtered. Combined with the signal of the plantar pressure sheet, the gait cycle was divided according to the pre-support, mid-support, end-support, and swing period. After filtering, five gait single-cycle sensor information graphs are extracted, as shown in Figure 10.

As shown in Figure 10, the square wave pattern is the sole pressure signal, the solid line is the forefoot pressure signal, and the dashed line is the heel pressure signal. Taking walking on flat ground as an example, the gyroscope signal is converted into an angle value according to the formula, and it can be seen from the comparison that the angle trend is consistent. Therefore, the sensor signal is reliable and effective and can reflect the basic situation of the human body when walking.

## 5. Gait Recognition

### 5.1. Differences in Plantar Pressure between Men and Women

Table 1 shows the statistical results of the peak plantar pressure of the male and female feet during walking.

As shown in Table 1, the peak plantar pressure distribution during walking has a greater change than the pressure distribution under the previous foot resting action. Each area of the foot plays a certain bearing role in the process of walking, and there are certain changes. The pressure distribution of male and female subjects was consistent, and the symmetry of the left and right feet was better. The statistical results of the peak plantar pressure of standing on one foot with eyes closed and standing on both feet of men and women are shown in Table 2.

As shown in Table 2, the sample data after preprocessing is divided into training samples and test samples. For the static data of 35 people, 10 stable frames are selected from the left and right foot plantar pressure image sequences as training samples and 3 frames as test samples. For the dynamic data of 35 people, from the left and right foot data of 10 walks at three different speeds, 7 frames of plantar pressure images with the largest plantar pressure value were selected as training samples, and 3 frames of plantar pressure were used as training samples. The plantar pressure image with the highest value is the test sample. The samples in static and dynamic situations are used as the input of the convolutional neural network, respectively, and the respective convolutional feature maps are obtained.

### 5.2. Gait Recognition Accuracy

The classifier is trained with the feature vectors obtained from the training samples of static data and dynamic data, respectively, and the classification results of the test samples are obtained. First, it experimented with the method on a static database. The plantar image area division uses three methods: four-area, eight-area, and this paper divides the sole of the foot into three areas and counts the pressure value of each area to obtain the area weight (called statistical three-area). The recognition accuracy obtained by different area division methods is shown in Table 3.

Table 3 shows the identification results of the experiment on the left foot pressure data of 35 people in the static database. It can be seen from the table that although the four-area and eight-area division methods reflect the plantar structure characteristics of people to a certain extent and achieve a recognition accuracy of more than 0.8 in the classification and recognition, their stability is not high enough. The recognition effect also needs to be further improved. The statistical three-region method proposed in this paper obtains higher recognition accuracy than the above two algorithms. This is because when calculating the features of R-CNN, it considers the size of the action of each region and assigns corresponding weights to each region. This greatly increases the effectiveness of the features and improves the final recognition results. In order to further illustrate the effectiveness of this area division method, the data of left and right feet at three different speeds of 35 people standing, walking, and standing on one foot with eyes closed were selected for experiments on the dynamic database. The identification results are shown in Table 4.

As shown in Table 4, during the dynamic data experiment, three experiments were performed on the left and right feet at each speed. It takes the average of the three results to obtain the average recognition accuracy at different speeds. It can be seen that when the plantar area is divided in advance and the weight of each area is marked, good recognition results can be achieved whether standing, walking, or standing with one leg closed, and the accuracy rate is above 90%. In comparison, slow walking is better than fast walking, and normal speed is in between. Therefore, gait recognition based on FCM model is also effective for dynamic data in static data domain, and it is a valuable gait recognition method.

The method of dividing the sole of the foot into eight regions to select features is used as the comparison algorithm in this paper to conduct experiments. The experimental data set is the plantar pressure information of 30 people in the dynamic database when they walk at three different speeds: normal speed, fast speed, and slow speed. The plantar pressure data collected at each different speed were carried out in three experiments according to different methods. The average of the three experimental results is shown in Table 5.

As can be seen fromTable 5, whether it is divided into four regions and eight regions to extract features or use the FCM model proposed in this paper for feature learning, the gait data obtained when walking at three different speeds are all different. The plantar pressure information collected when standing is the best, and the one-legged standing is the worst; this may be because the plantar pressure information collected when standing is more stable than standing on one foot and can better represent the distribution of plantar pressure. Therefore, the recognition accuracy rate is relatively high. At each speed, such as the experimental results of the plantar pressure data collected when walking at a normal speed, the average recognition accuracy of the FCM model proposed in this paper is above 90% for both the left foot and the right foot. The average accuracy rate is only about 80%, and the recognition accuracy rate using the method of dividing eight regions is 82%. It can be seen that the features extracted by the FCM model proposed in this paper contain more information of the plantar pressure image, and the accuracy rate is higher in classification and recognition.

## 6. Conclusion

Vision-based gait recognition is easily interfered by factors, such as environment and perspective. Haptic-based gait recognition is less susceptible to interference from external factors, but it is in its infancy. The features that characterize gait are not perfect, resulting in a low recognition rate. Therefore, a gait recognition algorithm based on the fusion of lower extremity joint angles and plantar pressure distribution features is proposed. In this paper, the lower limb joint angle and plantar pressure distribution features are fused in the feature layer, which improves the recognition rate. It performs periodic analysis of gait motion using the ratio of the width and height of the human side profile. In order to remove redundant frames, reduce feature dimensions, and improve computing speed, keyframe extraction is performed on gait, and lower limb joint angle features and plantar pressure distribution features are extracted respectively. It uses anatomical knowledge to automatically locate the joint points of human lower limbs in key frame images and extracts the joint angles of the lower limbs as visual features of gait. In the process of collecting the foot attitude information, the noise interference of the acceleration signal and the drift of the gyroscope signal affect the accuracy of the measurement. In this way, in the stage of foot horizontal support, there is always a small angle error between the detected foot posture pitch angle and the horizontal plane. However, the fusion of visual information and tactile information needs to be studied in depth to extract features that can better characterize the nature of gait.

## Figures and Tables

**Figure 1:** Common biological features.

**Figure 2:** The general process of tactile gait recognition.

**Figure 3:** Schematic diagram of a complete gait cycle.

**Figure 4:** The cross-correlation coefficients of the joint movements of the left and right legs.

**Figure 5:** Multisensor foot pressure acquisition signal.

**Figure 6:** Three-joint angles of hip, knee, and ankle.

**Figure 7:** Joint angles of walking on level ground, descending stairs, and descending slope gait. (a) Three-joint angle for level walking. (b) Three-joint angle for descending stairs. (c) Downhill three-joint angle.

**Figure 8:** Joint angles in stair-climbing and hill-climbing gaits. (a) Uphill three-joint angle uphill. (b) three-joint angle.

**Figure 9:** Plantar pressure signal normalized and divided into gait cycle.

**Figure 10:** Signal diagrams after filtering for five gaits. (a) Walking on level. (b) Down the stairs. (c) Downhill.

**Table 1:** Statistical results of peak pressure in each region of male and female subjects during walking.

Gender		H	T2-3	T4-5	MI	M2
Male	Left	1.261 ± 0.364	0.564 ± 0.143	0.346 ± 0.189	1.013 ± 0.279	2.046 ± 0.464
	Right	1.067 ± 0.413	0.561 ± 0.146	0.321 ± 0.156	0.946 ± 0.312	1.943 ± 0.167

Female	Left	1.179 ± 0.364	0.764 ± 0.146	0.279 ± 0.313	1.346 ± 0.464	2.246 ± 0.646
	Right	1.115 ± 0.246	0.615 ± 0.243	0.346 ± 0.264	1.067 ± 0.331	1.946 ± 0.346

**Table 2:** Statistical results of peak pressure in each region of male and female subjects standing on one foot with eyes closed and standing on one foot.

Gender		H	T2-3	T4-5	MI	M2
Male	Left	0.545 ± 0.286	0.265 ± 0.635	0.076 ± 0.146	0.695 ± 0.156	0.864 ± 0.081
	Right	0.556 ± 0.123	0.254 ± 0.152	0.035 ± 0.084	0.672 ± 0.145	0.816 ± 0.105

Female	Left	0.756 ± 0.265	0.356 ± 0.251	0.047 ± 0.068	0.876 ± 0.264	0.997 ± 0.167
	Right	0.55 ± 0.256	0.359 ± 0.265	0.032 ± 0.053	0.734 ± 0.246	0.881 ± 0.164

**Table 3:** Recognition accuracy obtained by different area division methods.

Recognition methods	Test 1	Test 2	Test 3
Stand	0.88	0.86	0.90
Walk	0.84	0.88	0.87
Stand on one foot with eyes closed	0.90	0.98	0.94

**Table 4:** Dynamic gait recognition accuracy.

Recognition methods	Left foot recognition accuracy				Right foot recognition accuracy			
Normal speed	1st	2nd	3rd	Average	1st	2nd	3rd	Average
Stand	0.94	0.92	0.94	0.933	0.92	0.92	0.94	0.927
Walk	0.89	0.86	0.88	0.877	0.90	0.87	0.86	0.877
Stand on one foot with eyes closed	0.96	0.94	0.94	0.947	0.96	0.94	0.96	0.953

**Table 5:** Comparison of recognition accuracy.

Recognition methods	Left foot recognition accuracy			Right foot recognition accuracy		
	Four regions (%)	Eight regions (%)	FCM (%)	Four regions (%)	Eight regions (%)	FCM (%)
Stand	80	82	92	78	82	91
Walk	76	78	93	76	78	88
Stand on one foot with eyes closed	80	84	95	80	82	93

## Data Availability

Data sharing not applicable to this article as no datasets were generated or analyzed during the current study.
